# Immunogenicity and Efficacy of Intramuscular Replication-Defective and Subunit Vaccines against Herpes Simplex Virus Type 2 in the Mouse Genital Model

**DOI:** 10.1371/journal.pone.0046714

**Published:** 2012-10-11

**Authors:** Simon Delagrave, Hector Hernandez, Changhong Zhou, John F. Hamberger, Sophia T. Mundle, John Catalan, Simge Baloglu, Stephen F. Anderson, Joshua M. DiNapoli, Patricia Londoño-Hayes, Mark Parrington, Jeffrey Almond, Harry Kleanthous

**Affiliations:** Sanofi Pasteur, Discovery North America, Cambridge, Massachusetts, United States of America; Cincinnati Childrens Hospital Medical Center, United States of America

## Abstract

Herpes simplex virus type 2 (HSV-2) is a sexually transmitted virus that is highly prevalent worldwide, causing a range of symptoms that result in significant healthcare costs and human suffering. ACAM529 is a replication-defective vaccine candidate prepared by growing the previously described *dl*5-29 on a cell line appropriate for GMP manufacturing. This vaccine, when administered subcutaneously, was previously shown to protect mice from a lethal vaginal HSV-2 challenge and to afford better protection than adjuvanted glycoprotein D (gD) in guinea pigs. Here we show that ACAM529 given via the intramuscular route affords significantly greater immunogenicity and protection in comparison with subcutaneous administration in the mouse vaginal HSV-2 challenge model. Further, we describe a side-by-side comparison of intramuscular ACAM529 with a gD vaccine across a range of challenge virus doses. While differences in protection against death are not significant, ACAM529 protects significantly better against mucosal infection, reducing peak challenge virus shedding at the highest challenge dose by over 500-fold versus 5-fold for gD. Over 27% (11/40) of ACAM529-immunized animals were protected from viral shedding while 2.5% (1/40) were protected by the gD vaccine. Similarly, 35% (7/20) of mice vaccinated with ACAM529 were protected from infection of their dorsal root ganglia while none of the gD-vaccinated mice were protected. These results indicate that measuring infection of the vaginal mucosa and of dorsal root ganglia over a range of challenge doses is more sensitive than evaluating survival at a single challenge dose as a means of directly comparing vaccine efficacy in the mouse vaginal challenge model. The data also support further investigation of ACAM529 for prophylaxis in human subjects.

## Introduction

HSV-2 is a global health problem, causing clinical manifestations ranging from mild skin or mucosal ulcers to lethal disseminated infections in newborns [1], [2]. According to a meta-analysis of seroprevalence surveys, over 530 million of 15 to 49-year-olds are infected, and more than 24 million new infections occur each year worldwide [3]. The health economic costs of HSV-2 infections have been projected to reach over $2.5 billion annually in the US alone by 2015 [4]. In an effort to address the medical and societal burden caused by HSV-2, a number of vaccines have been evaluated in the clinic over the past decades [5]. Notably, a subunit vaccine made using recombinant glycoprotein D of HSV-2 (gD-2) strain G was shown to be well tolerated and immunogenic [6], and to achieve a disease reduction of 73% (P = 0.01) and a trend for reduction in infections of about 43% (P = 0.08) in women who were HSV-1 seronegative [7]; however, a larger clinical trial with a different target population failed to demonstrate efficacy against HSV-2 and significantly increased shedding frequency in vaccine recipients who became infected with HSV-2 [8].

New vaccines are constantly being investigated for HSV prophylaxis [9], including live attenuated [10]–[12], DNA [13], subunit [14], peptides [15], [16], and prime-boost [17]. An alternative approach is the replication-defective virus *dl*5-29 which was constructed by deleting the U_L_5 and U_L_29 genes of herpes simplex virus type 2 (HSV-2) [18]. When administered to mice or guinea pigs subcutaneously, *dl*5-29 induces robust protective immune responses in vivo, and yet does not replicate or establish latency [19]–[21]. These data suggest that *dl*5-29 could be an effective vaccine for human use to prevent HSV-2 infections and genital herpes disease. In preparation for evaluation in a clinical setting, a new production cell line and virus master seed were prepared and the resulting vaccine was renamed ACAM529.

The replication-defective vaccine *dl*5-29 was previously shown in guinea pigs to be more immunogenic than purified subunit antigen gD combined with Freund's adjuvant, and, after vaginal challenge, to offer similar protection against disease while also significantly reducing shedding [20]. The vaccine was further shown to protect guinea pigs against latent infection regardless of whether they were previously infected with HSV-1 [21]. However, evaluation of the immunogenicity and efficacy of ACAM529, which is prepared using cells and virus seed intended for production of clinical trial material, had not been possible until recently. In addition, prior studies of efficacy were limited to a single challenge dose rather than a range of doses. Under these conditions, it was not possible to estimate by how much the vaccines increased the challenge dose required to infect a certain proportion of animals. This information may be useful in predicting clinical efficacy, particularly in light of the recent observation that gD did not protect against HSV-2 infection [8], which is consistent with past observations in guinea pigs [22].

Selection of immunization routes for human vaccines is highly empirical, however it is thought that immunization with live viral vaccines is less sensitive to route due to their ability to spread, while inactivated vaccines are generally most immunogenic when delivered intramuscularly or intradermally [23]. For instance, clinical studies have shown that delivery of measles, mumps, rubella, varicella combination vaccine (MMRV) is as effective by the intramuscular as the recommended subcutaneous route [24]. As a further example, delivery of live-attenuated polio vaccine is oral but the inactivated vaccine is given subcutaneously or intramuscularly. While the adjuvanted gD vaccine against HSV was given by intramuscular injection [7], the TA-HSV DISC vaccine, which was only tested for treatment of recurrent genital herpes but not prophylaxis, was administered subcutaneously [25]. The immunogenicity of *dl*29 (5BLacZ) via the intramuscular route was investigated previously [26], but its potency in a prophylactic challenge model has not been described, nor have the relative immunogenicity and protective efficacy of *dl*29 or *dl*5-29 delivered by the intradermal, subcutaneous and intramuscular routes. Mucosal delivery of *dl*5-29 via the intranasal route was reported, but only to show that the vaccine does not establish latency in trigeminal ganglia [19], and, interestingly, vaginal delivery of the vaccine in the guinea pig prophylactic model significantly reduced recurrent disease but the effect was inferior to that afforded by intramuscular gD, and intravaginal *dl*5-29 failed to reduce challenge virus loads in sacral ganglia, in contrast with gD [20].

In the present studies, we first investigate the optimal route for ACAM529 immunization against a vaginal challenge in mice. Then we compare the vaccine's efficacy with a glycoprotein D vaccine using four different challenge doses and several measures of immunogenicity and protection against viral infection as well as morbidity and mortality. These studies show that ACAM529 is most immunogenic and protective when given intramuscularly, and that it protects significantly better than gD against infection of the vaginal mucosa and dorsal root ganglia. Implications for preclinical assessment of vaccine candidates based on these observations are discussed.

## Results

### Immunogenicity and prophylactic efficacy of ACAM529 administered to mice via different routes

The effect of the route of administration of ACAM529 on its immunogenicity and protective efficacy was first investigated. BALB/c mice were immunized intradermally (ID), intramuscularly (IM), or subcutaneously (SC) and their blood sampled three weeks after the last vaccine dose. Serum prepared from this blood was tested for IgG responses against a commercial HSV-2 viral lysate (Fig. 1A), and assayed for neutralizing antibody responses (Fig. 1B). While all three immunization routes yielded significantly higher IgG responses compared to negative control animals, the IM group showed a significantly higher titer of 1.5×10^5^, nearly 10-fold higher than that shown by either the SC or ID groups. Neutralizing antibody responses observed in IM vaccinated mice were significantly higher than all other groups in the experiment, while the titers of SC and ID vaccinated mice were not significantly higher than the negative control group.

**Figure 1:** Characterization of antibody responses elicited by ACAM529 delivered via three different parenteral routes. Groups of ten BALB/c mice were immunized with two doses of 10^6^ pfu of ACAM529 given three weeks apart by one of three routes (SC, subcutaneous; IM, intramuscular; ID, intradermal), or with PBS (negative control given SC). Serum samples were taken 3 weeks after the second immunization. (A) ELISA endpoint IgG titers measured against whole HSV-2 lysate. Each symbol represents one animal and the horizontal bars indicate geometric mean titers (GMT). All differences except SC vs. ID are significant (* P<0.05; one way ANOVA, Kruskal-Wallis, Dunn's multiple comparison test). (B) Neutralizing antibody responses, reported as 50% plaque reduction neutralization titer (50% PRNT), are significantly higher in the IM group than in the SC or ID groups (*** P<0.0001; one way ANOVA). The dotted line indicates the lower limit of detection of the assay.

The mice were challenged intravaginally with 50 LD_50_ of HSV-2 strain 333 and their disease symptoms were monitored daily for two weeks. Animals that received the vaccine IM were 100% protected from challenge, which is significantly better than mice immunized SC (50% protection; P<0.02; Fig. 2A). ID immunization offered an intermediate degree of protection from death, and all three routes gave significant protection compared to mock immunization.

**Figure 2:** Effect of ACAM529 route of administration on prophylactic efficacy against a lethal challenge. Mice immunized as described in Fig. 1 were treated with medroxyprogesterone three weeks after the second immunization and challenged i.vag. one week later with 50 LD_50_ (8×10^4^ pfu) of HSV-2 strain 333. (A) The percentage of animals surviving the challenge is plotted as a function of days post-challenge. Survival of IM-immunized animals is significantly better than SC (* P<0.02). All three groups of immunized animals are significantly protected compared to mock-immunized (PBS) animals. (B) Two days after challenge, vaginal swabs were taken from all challenged animals and viral titers determined by plaque assay. Shed virus is significantly reduced in all groups compared to mock-immunized (PBS) animals, and IM-immunized animals shed significantly less compared to SC and ID (* P<0.05; one way ANOVA). One animal in the IM group died during a bleed, prior to challenge. The dotted line indicates the lower detection limit of the plaque assay.

Because survival from a lethal challenge is not considered to be a stringent measure of protection in the HSV-2 vaginal challenge model, we evaluated other metrics of infection. Shedding of challenge virus at the site of infection within two days of challenge is thought to be an indication of the extent of mucosal infection [22]. Using vaginal swabs, it is possible to measure the amount of virus shed into the vaginal cavity. Based on previous experiments (data not shown) it was established that the peak time of shedding is 48 hours (day 2) post-challenge. Therefore, the challenged animals were swabbed on the 2^nd^ day after challenge and the harvested virus titer was determined by plaque assay (Fig. 2B). All immunization routes afforded significant reductions in virus shedding compared to negative control animals, but IM immunization gave over 10-fold greater reduction in shed virus relative to SC or ID immunization (P<0.05). Interestingly, three of the IM mice and one of the ID mice had no virus detectable by plaque assay in their swabs, suggesting complete protection from mucosal infection.

### Comparison of the immunogenicity of ACAM529 and adjuvanted gD in mice

Having established the optimal delivery route for ACAM529, we wished to compare the immunogenicity and efficacy of ACAM529 and HSV-2 gD adjuvanted with CpG and alum [14], [27]. Two doses of 1×10^6^ plaque forming units (pfu) of ACAM529 were administered three weeks apart in the upper thigh, while three doses of 2 µg of adjuvanted gD were given two weeks apart in the gastrocnemius muscle as described previously [14]. Control animals received PBS SC, and all animals received the last vaccine dose on the same day. The animals were bled 10 days after the last dose and sera were assayed for neutralizing antibody titers (Fig. 3A), IgG against HSV-2 lysate (Fig. 3B), as well as IgG against purified recombinant gD (Fig. 3C). Both ACAM529 and gD elicited similar neutralizing antibody titers against HSV-2, and while ACAM529 gave a 16-fold higher IgG titer against HSV-2 lysate than gD, gD-immunized mice showed a 14-fold greater titer against purified gD than ACAM529-immunized mice (both differences statistically significant).

**Figure 3:** Comparison of the immune responses to ACAM529 and gD in mice. Groups of 60 female BALB/c mice received either two doses given three weeks apart of 10^6^ PFU of ACAM529, or three doses given two weeks apart of gD (2 µg adjuvanted with CpG and alum), or PBS, all given IM. The last dose was received on the same day for all groups. Serum was collected nine days after the last dose. (A) Plaque reduction neutralization titer (50% PRNT) in the presence of complement. The vaccine groups are significantly higher than PBS and not significantly different from each other (one way ANOVA). (B) Total IgG ELISA against HSV-2 lysate. All 3 groups are significantly different from each other (* P<0.05; one way ANOVA). (C) IgG endpoint titers determined by ELISA against purified recombinant gD for mice immunized with ACAM529 or gD. Immunization with gD gave significantly higher anti-gD titers than immunization with ACAM529 (*** P<0.0001; two-tailed t test). (D) In parallel with the larger groups of mice discussed above, three groups of six mice were immunized in the same way and their spleens harvested 9 days after the last vaccine dose. Splenocytes were cultured in the presence of the I-A^d^-restricted CD4+ T cell epitope represented by gD-2 peptide 245–259, and HSV-specific CD4+ T cell responses were quantitated based on the frequency of interferon-γ-secreting cells following stimulation. The indicated values represent the mean for each group calculated based on triplicate measurements made for each splenocyte sample and error bars indicate the standard error for the group. ACAM529 is significantly different from both the gD and PBS groups (* P<0.05; one way ANOVA). The dotted line indicates the detection limit in (A) and (B) above.

An interferon-γ ELISPOT was carried out on a subset of immunized animals whose spleens were harvested 9 days after the last vaccine dose. Splenocytes were cultured in the presence of an immunodominant I-A^d^-restricted gD peptide and interferon-γ-secreting cells were counted. The CD4+ T cell response of ACAM529-immunized animals is significantly greater than that seen in gD-immunized mice or negative control mice (Fig. 3D). Similar results were obtained using UV-inactivated ACAM529 for stimulation of splenocytes in the ELISPOT (data not shown).

### Comparison of the prophylactic efficacy of ACAM529 and adjuvanted gD in mice

The immunized animals were challenged with wildtype HSV-2 to compare the efficacy of the two vaccines, however, in order to increase the probability of finding conditions which would reveal any differences, the animals were given one of four different challenge doses. Eleven days after the last vaccine dose, the immunized mice were given 2 mg of medroxyprogesterone and challenged intravaginally 7 days later with one of four challenge doses of HSV-2 strain 333: 15 LD_50_ (2.4×10^4^ pfu), 50 LD_50_ (8×10^4^ pfu), 150 LD_50_ (2.4×10^5^ pfu), or 450 LD_50_ (7.2×10^5^ pfu). For two weeks following challenge, the animals were observed for morbidity and mortality.

The effect of immunization on disease severity is shown in Fig. 4A. Control animals experienced significantly more severe symptoms than immunized mice at all challenge doses. ACAM529 protected mice significantly better than gD at all challenge doses tested. Animals reaching a disease score of 3 or higher were euthanized in accordance with approved institutional animal care protocols. All mock-immunized mice died or were euthanized by day 9 post-challenge (Fig. 4B and not shown). While four of forty mice were euthanized in the gD-immunized group, none of the ACAM529-immunized animals died or required euthanasia, although this was not a statistically significant difference (Fig. 4C; Fisher's exact test, P = 0.12).

**Figure 4:** Morbidity and mortality of immunized mice challenged with a range of wildtype HSV-2 doses. Mice immunized as described in Fig. 3 were treated with medroxyprogesterone, divided into 4 challenge groups of 10 animals each, and challenged intravaginally 19 days after the last vaccination with either 15, 50, 150 or 450 LD_50_ of HSV-2 strain 333. (A) Morbidity was observed for two weeks following the challenge and is plotted here as the mean disease score averaged over the entire observation period, with error bars indicating standard error. ACAM529 significantly reduced morbidity at all challenge dose levels as compared to PBS and gD (P<0.05). (B) Survival of immunized mice challenged with 50 LD_50_ of HSV-2 is plotted as a function of days post-challenge. Differences between both groups and PBS are statistically significant, but there is no significant difference between ACAM529 and gD. (C) Survival at the end of the two-week observation period is plotted as a function of challenge dose for mock (PBS), ACAM529, and gD-immunized mice. Vaccination gave significant protection against mortality at all challenge doses compared to mock-immunization (PBS), but differences between the two vaccines were not significant.

Mucosal replication of challenge virus was measured by taking vaginal swabs of the mice during peak shedding (day 2 post-challenge) and measuring swab viral titers by plaque assay. The observed shedding for animals challenged with the highest dose is shown in Fig. 5A. ACAM529 significantly reduced shedding from 1.9×10^5^ pfu (geometric mean) for mock-immunized mice to 3.2×10^2^ pfu, which is a statistically significant decrease of over 500-fold. Furthermore, two of ten ACAM529-immunized animals had non-detectable shedding. Immunization with gD afforded a non-significant 5-fold decrease in shedding at this challenge dose.

**Figure 5:** Protection against mucosal infection as measured by plaque assay of vaginal swabs. Animals described in Fig. 4 were swabbed intravaginally on day 2 post-challenge and the shed virus titers determined by plaque assay. (A) Shedding for animals challenged with 7.2×10^5^ PFU (450 LD_50_) of wildtype HSV-2 (one symbol per mouse). ACAM529 significantly reduced viral shedding compared to gD, and only ACAM529 is significantly better than PBS (* P<0.05; one way ANOVA). (B) Virus shedding is plotted as a function of the challenge dose. ACAM529 significantly reduces virus shedding compared to mock-immunized (PBS) animals at all doses tested while gD affords significant protection at the lowest challenge dose (* P<0.05 compared to PBS; one way ANOVA). (C) Protection from peak virus shedding. The percentage of mice for which shedding was below the detection limit on day 2 is plotted as a function of decreasing challenge dose. Overall, more animals were protected by ACAM529 than gD (P = 0.0033; Fisher's exact test).

Figure 5B shows the amount of virus shed as a function of challenge dose for mock-immunized, ACAM529-immunized, or gD-immunized animals. Mock-immunized mice shed increasing amounts of virus with increasing challenge dose and reached a plateau at the 2.4×10^5^ pfu dose. There was a similar trend observed for gD-immunized mice, except that there was significant reduction in shedding observed at the lowest challenge dose. ACAM529 afforded significant reductions in shedding compared to control mice at all challenge doses.

The proportion of mice protected from challenge, i.e., with plaque titers below the detection limit, was also analyzed (Fig. 5C). At all four challenge doses, ACAM529 protected 20% to 40% of animals from shedding, while protection was only observed in one animal (10%) immunized with gD at the lowest challenge dose. Overall, combining all challenge dose groups, 27.5% (11/40) of ACAM529-immunized animals were protected from viral shedding while 2.5% (1/40) were protected by the gD vaccine (P = 0.0033; Fisher's exact test).

Protection against infection of the dorsal root ganglia (DRG) was done in a subset of animals which was challenged 58 days after the last vaccine dose. Four days after challenge, five pairs of DRG were extracted from each mouse and their DNA extracted in order to carry out quantitative PCR to measure viral genome copy number. The number of viral genome copies was divided by copy number of the host gene adipsin and this ratio is plotted in Fig. 6A for all four challenge doses. Both the ACAM529 and gD vaccines significantly reduce DRG viral DNA loads compared to negative control mice. The proportion of animals with undetectable viral genomes, i.e., protected from DRG infection, is shown in Fig. 6B. Overall, 7 of 20 mice (35%) are protected by ACAM529, while none of the gD-immunized mice were protected (P = 0.0083; Fisher's exact test).

**Figure 6:** Protection against infection in dorsal root ganglia. A subset of the animals immunized as described in Fig. 3 was challenged intravaginally, as described in Fig. 4, 58 days after the last vaccine dose, and dorsal root ganglia were extracted 4 days post-challenge. Viral genome copies in ganglia were determined by quantitative PCR and reported as a ratio with the host gene adipsin. (A) Viral DNA loads in dorsal root ganglia are significantly reduced by immunization. (P<0.05, one way ANOVA, Tukey's comparison. Twenty animals in each group were divided in to 4 groups of 5 animals for each challenge dose. To permit GMT calculation, samples with undetectable viral genome copies were increased from 0 to 0.1. Error bars indicate standard error of the mean.) (B) Protection from infection of dorsal root ganglia. The percentage of mice for which viral genome copies in DRG were below the detection limit on day 4 is plotted as a function of challenge dose. ACAM529 consistently protects ≥20% of mice from DRG viral infection (n = 5). Combining mice at all challenge doses, ACAM529 protected more mice than gD (P = 0.0083; Fisher's exact test).

## Discussion

According to Belshe et al. [8], gD-2 adjuvanted with alum and 3-O-deacetylated MPL protected women against HSV-1 infection and disease but did not protect them from HSV-2. Instead, it caused a significant increase in virus shedding frequency among vaccine recipients who became infected with HSV-2. This suggests that new vaccines based on different antigens and exploiting different antigen presentation mechanisms, must be investigated to eventually achieve the goal of effective prophylactic immunization against this virus. Therefore, preclinical evaluation of vaccine candidates is important in prioritizing resources for future clinical studies, and the efficacy of gD serves as a benchmark which must be exceeded for a vaccine to go forward into clinical development.

An important consideration in the development of ACAM529 was the ideal route of immunization. Past studies generally evaluated SC delivery both in mice and guinea pigs [18], [20], however Figs. 1 and 2, as well as unpublished results (not shown) obtained in our laboratories with a lower dose of the vaccine, indicate superior immunogenicity and efficacy of ACAM529 when it is administered IM. While the greater anatomical proximity of the IM injection (in the upper thigh) to the challenge site (intravaginal) might help increase efficacy as compared to SC injections (scruff of neck), this would not explain the significantly higher antibody titers elicited when the vaccine is given by the IM route. This suggests that the increased prophylactic effect is unlikely to be due to the anatomical proximity of immunization and challenge sites. The same logic applies to the ID injections in the flank of the mice, which were no more immunogenic or efficacious than SC. Recently, Awasthi et al. also reported a trend for intramuscular administration of their HSV-2 gE-deletion mutant vaccine to be more effective against shedding and disease than subcutaneous immunization in mice [28].

Past studies of gD adjuvanted with MPL and alum [22] have shown that protection against mucosal infection in guinea pigs is not achieved with this vaccine despite nearly complete prevention of morbidity and mortality. Therefore it is important to consider more than symptoms of disease when assessing vaccine efficacy. In addition, it is currently very difficult to conclusively compare vaccines using published data due to the variety of challenge strains being used that have different passage histories and apparently different virulence, as well as other differences in infection protocols, animal model used, immunological protocols, virological assays, etc. These considerations militate in favor of side-by-side comparisons of vaccines against HSV-2 with a benchmark immunogen such as adjuvanted gD.

In this study, ACAM529 was compared with gD combined with alum and CpG adjuvant as described by Awasthi et al. [14]. A similar vaccine was recently evaluated by Khodai et al. [29] and found to be more immunogenic than gD adjuvanted with MPL and alum. Because we were interested in finding conditions that optimally differentiate ACAM529 and gD, we challenged groups of immunized animals with different doses of wildtype HSV-2, spanning a 30-fold range from 15 to 450 LD_50_ (2.4×10^4^ to 7.2×10^5^ pfu). Based on our past experience we doubted that even a severe challenge would be enough to differentiate the two vaccines and this was borne out by the lack of significant differences in mortality, although disease symptoms were significantly lower in ACAM529-immunized mice as compared to gD.

Among mice immunized with gD, there was a trend for mean disease scores to increase with challenge dose until the highest dose, at which point the mean disease score decreased slightly, but these differences were not significant. Also in the gD recipients, more deaths were seen in the 50 LD_50_ group than the 150 or 450 LD_50_ groups, however these differences are not statistically significant and are consistent with the expectation that gD achieves a protection against morbidity and mortality that is robust enough to render these metrics unhelpful in comparing different vaccines.

Mucosal infection can be assessed by measuring challenge virus shedding using vaginal swabs within the first two days post-challenge [22]. Similarly, measuring viral genome copy number in DRG indicates the extent to which the infection has spread to sensory ganglia. ACAM529 achieved significantly greater reductions in mucosal replication (Fig. 5A and B). In addition, ACAM529 achieved significant protection against both mucosal and DRG infection while gD did not (Figs. 5C and 6B). A further benefit of challenging with a range of doses is that the effect of immunization on the dose of challenge virus leading to 90% infection (ID90, or Infectious Dose 90%) can be estimated. While 90% of gD-vaccinated mice could be infected with the lowest challenge dose, the dose required to infect the same proportion of ACAM529-vaccinated mice was not reached in this study. Therefore, ACAM529 vaccination increases the ID90 by more than 30-fold over gD vaccination. The shift in ID90 relative to mock immunization cannot be estimated because 100% of mice were infected even at the lowest challenge dose.

These differences in efficacy cannot be explained by differences in the neutralizing antibody responses since the titers induced by either vaccine were not significantly different (Fig. 3A). Also, antibody titers against gD are significantly higher in gD-immunized animals compared to those that received ACAM529, as might be expected given the compositions of the vaccines (Fig. 3C). These two observations, along with the observations mentioned earlier of significant protection against morbidity and mortality, are also consistent with a successful immunization with gD. In contrast, antibody titers measured by ELISA against an HSV-2 lysate are significantly higher in the group of animals which received the vaccine that comprises multiple HSV-2 antigens, namely ACAM529 (Fig. 3B). Moreover, interferon-γ ELISPOT data acquired by stimulation of splenocytes with a gD peptide known to stimulate CD4+ T cells indicate a significantly greater response in mice immunized with ACAM529 (Fig. 3D). Therefore, both total anti-HSV-2 IgG responses and CD4+ interferon-γ+ T cell counts correlate with protection in this study. The latter observation is consistent with past reports of the importance of CD4+ T cells in mice to achieve robust prophylaxis [30], [31]. These data indicate that there are qualitative differences in the obtained immune responses which lead to differences in protective efficacy.

## Conclusion

The observations reported here support the proposition that intramuscular immunization with ACAM529 should be investigated in clinical studies. Moreover, we propose that preclinical evaluation of future vaccine candidates should include a benchmark vaccine such as adjuvanted gD, and should measure protection against mucosal and DRG infection in addition to morbidity and mortality, preferably with a publically available reference challenge strain. Other methods of standardization may further accelerate the search for a potent prophylactic HSV-2 vaccine and should be considered by researchers in the field. Finally, new ex vivo human models of immunogenicity should be considered as a potentially rich new source of information to compare and optimize human HSV vaccines [32].

## Materials and Methods

### Complementing cells

Complementing cell line AV529-19 was obtained by combining the Vero cell line CCL-81.2 (ATCC, Manassas, VA) with plasmids pCId.UL5, pcDNA.UL29, and pSV2neo, which were provided by Dr. David Knipe (Harvard Medical School). To minimize the chance of homologous recombination between the transgenes and the vaccine genome during manufacturing, all flanking sequences of the HSV-1 U_L_5 and U_L_29 genes were removed before cloning except for a 109 bp segment in the 3′ untranslated region of U _L_5 sharing 72% identity with the vaccine genome. The transfected cells were cloned and screened for their ability to complement *dl*5-29. Despite repeated passaging of ACAM529 in vitro, replication-competent virus has never been observed (data not shown). The cells were maintained in OptiPro (Invitrogen, Carlsbad, CA) supplemented with 10% FBS (Hyclone, Logan, UT) and 4 mM glutamine (Invitrogen) at 37°C in a 5% CO_2_ atmosphere.

### Viruses

Viral genomic DNA encoding vaccine virus *dl*5-29 was provided by Dr. David Knipe (Harvard Medical School). To produce the pre-master seed, this DNA was transfected into AV529-19 and the resulting virus was passaged once to amplify titers. Viral genomic DNA was extracted from this virus passage and used to transfect AV529-19 again under GLP conditions. The resulting virus was harvested, plaque-purified four times, and banked under GMP. The selected clone is identified as ACAM529 clone 4a. Vaccine utilized for *in vivo* studies was purified in a process to be described elsewhere (Mundle et al., *in preparation*).

HSV-2 challenge strain 333 was a generous gift of Dr. Jeffrey Cohen (NIAID, Medical Virology Section). Challenge virus was cultivated on Vero cells seeded one day before infection at 1.2×10^7^ cells in T175 flasks. Virus was inoculated at a multiplicity of infection of 0.01 pfu/cell. Flasks were incubated at 37°C, 5% CO_2_ for 1 h with agitation every 15 minutes. After addition of 20 mL of fresh media (DMEM containing 1% FBS), cultures were allowed to incubate under the same conditions until 100% cell death was reached (about 2 days). Infected cells were harvested and lysed to extract the virus.

### gD vaccine

Recombinant HSV-2 glycoprotein D comprising residues 1–306 was produced in baculovirus and provided by Dr. Gary H. Cohen (Department of Microbiology, School of Dental Medicine, University of Pennsylvania) [14], [27]. The antigen (gD, 2 µg/mouse) was mixed with CpG oligonucleotide ODN1826 (50 µg/mouse; InVivogen, CA) and with alum (25 µg/mouse; Alhydrogel, Accurate Chemicals and Scientific Corporation, MO) and combined using a vortex mixer for 2 hours at room temperature before injection.

### Plaque assays

Samples were serially diluted and plated onto 12-well plates seeded one day prior to inoculation with 4×10^5^ AV529 cells per well. Plates were incubated at 37°C, 5% CO_2_ for 1 hour with gentle rocking of plates every 15 min. Overlay medium (1 mL) consisting of methyl cellulose in DMEM supplemented with heat-inactivated FBS, L-glutamine and antibiotics was then added to each well. Plates were incubated at 37°C, 5% CO_2_ for about 48 hours. Following incubation, plates were stained with 1% crystal violet in 70% methanol. Plaques were then counted and titers calculated in pfu/mL.

### Ethics statement

All animal experiments were performed according to Animal Research Protocol number 2011-05-01 approved by Sanofi Pasteur's Institutional Animal Care and Use Committee, Acambis Cambridge Campus.

### Mouse challenge model

Female BALB/c mice 6–7 weeks old were purchased from Charles River (Wilmington, MA). Animals were vaccinated with 1×10^6^ pfu ACAM529 in 100 µL of sterile PBS. In the first route study, control animals were inoculated subcutaneously with sterile PBS, while in the gD comparison study, all control animals were immunized intramuscularly in the heavy musculature of the upper thigh. Subcutaneous immunization was administered in the scruff of the neck. Intramuscular immunization of 100 µL of ACAM529 was given in the upper thigh using a 27G needle. Intramuscular immunization with gD was in the gastrocnemius. Intradermal administration was done by first wiping the animal with 70% ethanol, then the skin of the back was pulled taut with one hand and the 27G needle was injected bevel up at a shallow angle and two injections of 50 µl were given per mouse. Serum samples for serology assays were obtained from mandibular bleeds.

Seven days prior to intravaginal (i.vag.) challenge, mice were injected subcutaneously with 2 mg of medroxyprogesterone acetate injectable suspension diluted in PBS (SICOR Pharmaceuticals Inc., Irvine, CA). On the day of challenge, mice were given, in the route comparison experiment, 50 LD_50_ (8×10^4^ pfu), and in the gD comparison experiment 15, 50, 150 or 450 LD_50_ of HSV-2 strain 333 i.vag. in 20 µL sterile PBS with a positive displacement pipette. Pathology was scored on a 4 point scale as follows: 0 = no signs of disease, 1 = slight genital erythema and edema; 2 = moderate genital lesion and/or loss of fur; 3 = purulent genital lesion; 4 = hind-limb paralysis. Mice were euthanized upon reaching stage 3 or 4. Animals were observed and disease scores were recorded daily for 14 days after challenge.

### Vaginal swabs

Vaginal swabs were taken on day two after challenge, and in some cases on days one, four and/or six, using swabs (CleanTips Swab, Micro CleanFoam Head, ITW Texwipe). Swabs were collected in 1 mL stabilization buffer and stored at −80°C until challenge virus titers were determined by plaque assay.

### ELISAs

ELISA against HSV-2 lysate was performed using Maxisorp plates (Nunc) which were coated with 100 µl/well of a solution of 2 µg/ml of HSV-2 purified viral lysate in PBS (Advanced Biotechnologies). Serum IgG was detected with biotin-anti-mouse IgG (Fc) (Sigma) diluted 1∶2000 in 1% BSA/0.05% Tween 20 in PBS which was measured by time resolved fluorescence (TRF) using the Victor II fluorometer (Perkin Elmer) by adding Delfia europium–streptavidin conjugate at a concentration of 0.1 µg/ml in Delfia Assay Buffer.

The ELISA against gD was carried out according to the same protocol as the HSV-2 lysate ELISA protocol except that plates were coated with soluble recombinant gD-2 from HSV-2 using 100 µl/well of a solution of 0.5 µg/mL of gD-2 in PBS.

### Virus neutralization assay

Serum neutralizing antibodies were measured by pre-incubating serum dilutions with HSV-2 strain 333 and plating the mixture over AV529-19 cells for an hour. The resulting assay plates were incubated 2 days at 37°C, 5% CO_2_, and fixed and stained using a crystal violet methanol solution. Neutralizing titer was defined as the highest dilution of the serum to reduce the average pfu/well by ≥50% from the average pfu number in the negative controls. In the route comparison experiment, complement was not added to the assay, while in the gD comparison guinea pig serum (Calbiochem) was added to a final concentration of 5%.

### ELISPOT

Prior to animal sacrifice, opaque 96-well tissue culture plates (Millipore) were coated with 0.5 µg per well of anti-mouse interferon-γ antibody (BD Biosciences) and then incubated at room temperature for 2 hours. The coating antibody was then discarded and the wells were blocked with complete RPMI containing 10% fetal bovine serum, 55 µM β-mercaptoethanol, and antibiotic/antimycotic (Invitrogen) for 2 hours at room temperature. To obtain splenocytes from experimental animals, mice were sacrificed by CO_2_ asphyxiation and the spleens were harvested and placed in complete RPMI medium. Each organ was ground through a cell strainer (BD Biosciences) using a syringe plunger and the resulting cell pellet was incubated in red blood cell lysis buffer (Sigma Aldrich) for 2 to 3 minutes followed by extensive washing with complete RPMI medium. The coated tissue culture plates then received 2×10^5^ live splenocytes per well and a stimulation mixture containing either concanavalin A at 2.5 µg/mL, HSV gD-2 peptide 245–259 at 10 µg/mL, UV-inactivated ACAM529 at 10^6^ PFU/mL, or medium alone for mock stimulation, in a final volume of 200 µL per well. Each condition was tested in triplicate for each splenocyte sample. Following cell stimulation at 37°C for 20 hours, wells were washed and sequentially incubated with biotinylated anti-mouse interferon-γ (BD Biosciences) at 2 µg/mL, alkaline phosphatase-conjugated streptavidin (Jackson Immunoresearch) at 1 µg/mL, and then BCIP/NBT phosphatase substrate (Sigma Aldrich) as per the manufacturer's directions. Spots were counted using a CTL-ImmunoSpot S5 UV Analyzer (Cellular Technologies Limited) and the value for each splenocyte sample was reported as the mean number of spots per 10^6^ cells from triplicate wells.

### Quantification of viral load in DRG

Dorsal root ganglia (DRG) were dissected according to Malin et al. [33], frozen at −80°C in DMEM containing 5% FBS as well as antibiotics, and sent to Dr. Harvey Friedman (University of Pennsylvania) for analysis. DNA was extracted from mouse DRG samples and analyzed using duplex real-time qPCR to quantify the HSV-2 Us9 gene, with a previously reported limit of quantitation of 5 copies, and the mouse adipsin gene as described previously [14].
